The article "Comparison of Diagnosis Accuracy between a Backpropagation Artificial Neural Network Model and Linear Regression in Digestive Disease Patients: an Empirical Research" was published in 2021. Journal: Comput Math Methods Med.

# Comparison of Diagnosis Accuracy between a Backpropagation Artificial Neural Network Model and Linear Regression in Digestive Disease Patients: an Empirical Research

**DOI:** 10.1155/2021/6662779

**Published:** 2021-02-27

**Authors:** Wei Wei, Xu Yang

**Affiliations:** ^1^Clinical Epidemiology and Evidence-Based Medical Center, Beijing Friendship Hospital, Capital Medical University, National Clinical Research Center for Digestive Diseases, Beijing 100050, China; ^2^School of Computer Science and Technology, Beijing Institute of Technology, Beijing 100081, China

## Abstract

**Introduction:**

A Noninvasive diagnosis model for digestive diseases is the vital issue for the current clinical research. Our systematic review is aimed at demonstrating diagnosis accuracy between the BP-ANN algorithm and linear regression in digestive disease patients, including their activation function and data structure.

**Methods:**

We reported the systematic review according to the PRISMA guidelines. We searched related articles from seven electronic scholarly databases for comparison of the diagnosis accuracy focusing on BP-ANN and linear regression. The characteristics, patient number, input/output marker, diagnosis accuracy, and results/conclusions related to comparison were extracted independently based on inclusion criteria.

**Results:**

Nine articles met all the criteria and were enrolled in our review. Of those enrolled articles, the publishing year ranged from 1991 to 2017. The sample size ranged from 42 to 3222 digestive disease patients, and all of the patients showed comparable biomarkers between the BP-ANN algorithm and linear regression. According to our study, 8 literature demonstrated that the BP-ANN model is superior to linear regression in predicting the disease outcome based on AUROC results. One literature reported linear regression to be superior to BP-ANN for the early diagnosis of colorectal cancer.

**Conclusion:**

The BP-ANN algorithm and linear regression both had high capacity in fitting the diagnostic model and BP-ANN displayed more prediction accuracy for the noninvasive diagnosis model of digestive diseases. We compared the activation functions and data structure between BP-ANN and linear regression for fitting the diagnosis model, and the data suggested that BP-ANN was a comprehensive recommendation algorithm.

## 1. Introduction

Digestive disease involves the tube from the esophagus to the stomach and intestines as well as various organs connected to this tube such as the liver and pancreas, which are very complicated medical situations involving multiple-organ systems and biochemistry, immunology, and pathology mechanisms [1]. Based on the 2015 China Health Statistics Annuals, the two-week prevalence and chronic disease prevalence of digestive diseases were 15‰ and 24.9‰, respectively [2]. American Centers for Disease Control and Prevention (CDC) reported almost 60 to 70 million people being affected by all kinds of digestive diseases in 2001, and 9.3% (18.9 million) of noninstitutionalized adults were diagnosed with digestive disorders annually (Summary Health Statistics for US Adults, 2001, NCHS, CDC) [3]. Economists estimated $912,443,000 being spent in public hospitals on digestive system diseases in Australia from 2001 to 2002 (AIHW National Hospital Morbidity Database, Australia's Health 2004, AIHW) [4] (https://www.rightdiagnosis.com/d/digest/stats.htm). The five-year survival of most digestive diseases is more than 80% if patients could be diagnosed or treated at an early stage [5].

In a previous study, many researchers extracted noninvasive biomarkers for constructing diagnosis or a predictive model at an early disease stage in digestive disease patients, especially in tumors that have shown a great value for medical practice due to the rapid test and convenient sampling of these biomarkers [6]. WHO (World Health Organization) guidelines recommended that APRI and FIB-4 could be applied in HBV-reduced fibrosis assessment instead of invasive examinations in limited medical resource countries [7]. And the Lok score performed well in diagnosing portal hypertension using transient elastography (TE) [8]. Gurung et al. used AST/ALT (the AST-to-ALT ratio) to elevate in the alcoholic liver disease pattern in patients with hepatitis C who progressed to liver cirrhosis [9]. Lin et al. constructed the noninvasive diagnosis of nonalcoholic fatty liver disease and quantification of liver fat using a new quantitative ultrasound technique [10]. Characteristic information, hematological examination, biochemical detection, endoscopic ultrasonography, and pathology score were used in mathematical modeling to predict the disease outcome accurately [11–14]. A well-designed model can estimate the complicated, undefined relationship between risk factors as input biomarkers and the probability of occurrence of digestive disease as the output variable [15].

In the most common multivariate statistical model for diagnosis or prediction, biomarkers were extracted as dependent variables in order to derive the linear influence relationship between biomarkers and response variables [16–18]. However, these high-dimensional data collected from different visits were complicated for linear regression and collinearity between correlated biomarkers could not be detected or solved in the linear model [19]. A sophisticated artificial neural network (ANN) algorithm, the backpropagation ANN model, was able to construct vague and nonlinear connections between input biomarkers and the target biomarker through the simulation of complicated processing neurons. The correlation between input variables and target data could be learned by the ANN after training several times [20, 21]. The ANN model mimicked signal transmission in human brains through a set of processing units which consist of neurons, and these neurons were interconnected via the weight connections which make signal transmission in parallel and series [22–24]. The most representative construction of ANN consisted of three layers [25]. For clinicians and statisticians, the input layer represented the observed biomarkers of serum biochemical and auxiliary examinations [26, 27]. The output layer was the indicator of clinical outcomes. The processing of ANN was driven by input data, and the decision making was achieved with minimum adjustments by human [28–30]. In the modeling process, training data were analyzed and then the decision was made through output neurons when new input variables were put in [31]. In most of the ANN models, the backpropagation (BP) network was the commonly used solution in dealing with the nonlinear relationship between input variables and output variables by constantly adapting the connection weight value between neurons and the error threshold in each layer to make the output variables approximately towards the expected outcome [32–36]. The BP algorithm was based on error gradient descent (Figure 1), which was aimed at finding the minimum error by adjusting weights of connections between neurons in the direction of lowest error [37]. The error was estimated from the output variable and backcalculated to converge to the optimum solutions [38].

In linear regression, we assume that the input medical biomarkers and the clinical outcomes would be connected through a nonlinear link function. The BP algorithm demonstrates the modification of weights between synaptic neurons during learning, and the connection would be changed according to an error term computed for neurons throughout each layer. Each computed weight is corrected by the parameters of the activity of the neuron and the error term of the neuron it projects to. We could establish the complicated mathematical model between the input medical biomarkers and each matching output variables. In view of these benefits and limitations, the algorithm with a more accurate calculation and more concise demonstration would be the optimum solution for medical decision. However, the appropriate choice either linear regression or BP-ANN has not been reported in the recent publications and whether the BP-ANN algorithm is always more accurate versus linear regression is controversial. Therefore, our research will try to discuss the following questions based on a systematic review:

1. The characteristics of current studies using the BP-ANN algorithm and linear regression
2. The correlations between the BP-ANN algorithm and linear regression
3. Comparison of diagnosis accuracy between the BP-ANN algorithm and linear regression for digestive diseases

## 2. Methods

### 2.1. Correlations between the BP-ANN Algorithm and Linear Regression

In respect of linear principal component structure data, linear regression could be interpreted as a one-layer perceptron neural structure model, which included input variables and output variables (Figure 2). The input layer transmitted the input clinical biomarkers directly to the output variable through sigmoid function, which would calculate the weight of each input variable in linear regression, that is equal to the regression coefficient using the least square method [39, 40].

The activation function is a very important issue because it is the direct bridge between input variables and the clinical outcome, which greatly affect the prediction accuracy. According to the activation function, nonlinearity correlation would be transformed to linear regression, which is an effective solution for calculating the parameters in the hidden layer [41]. Different types of activation functions may lead to different neural network parameters, and the commonly used activation functions include the sigmoid function, tanh function, and Gaussian function [42–44].

(1) $$\begin{array}{c} h\left(x\right)=\frac{1}{1+e^{-\left(ax+b\right)}},\\ \tan h\left(x\right)=\frac{\sin h\left(x\right)}{\cos h\left(x\right)},\\ h\left(x\right)=e^{-{\left(x-\omega_{i}\right)}^{2}/\rho_{i}^{2}}. \end{array}$$

The input variables were fitted by linear regression before the activation function was applied, as shown in Figure 2, where Figures 2(a) and 2(b) represented the intercept and the coefficient, respectively. In the sigmoid function, variables transformed to the “*s*” curve and its value is between 0 and 1. In the tanh function, the value transformed between −1 and 1. In the Gaussian function, *ω*_*i*_ and *ρ*_*i*_ were the center and length, respectively. As seen in equation (1), the activation functions were complex for researchers to determine the optimal function because of the change of parameters; therefore, the machine learning algorithm is used to help optimize and fit an activation function for the neural network [45].

### 2.2. Error Propagation in BP-ANN and Linear Regression

The linear regression for principal component analysis fitted the straight line which crosses the hidden layer in the neural network, and the next process was to generalize this straight line to a curve. Based on the principal component analysis, the BP-ANN model could fix nonlinear principal component data and the algorithm was backpropagation for mean square error (MSE) and composed of a gradient descent method which was widely used in numerical minimization of a preestablished cost function [38, 46]. According to the gradient trends, the BP model could update parameters between hidden layers and the input layer [47]. Combined with the BP network structure, the process of error propagation started from the output layer as follows:

(2) $$\begin{array}{c} E=\underset{k}{\sum }E_{k}=\underset{k}{\sum }\frac{1}{2}{\left(d_{k}-o_{k}\right)}^{2}, \end{array}$$

where *E* is the total error and *E*_*k*_ is the error for the *k*^th^ output neuron, which is the deviation between the actual output *o*_*k*_ and expected output *d*_*k*_ of the *k*^th^ output neuron.

If the above error definition formula is extended to hidden layer neurons, where *y*_*j*_ represents the output of the *j*^th^ hidden layer neuron and *ω*_*jk*_ represents the weight of the connection between the *j*^th^ hidden layer neuron and the *k*^th^ output neuron, then

(3) $$\begin{array}{c} E=\underset{k}{\sum }E_{k}=\frac{1}{2}\underset{k}{\sum }{\left[d_{k}-o_{k}\right]}^{2}=\frac{1}{2}\underset{k}{\sum }{\left[d_{k}-f\left({\text{net}}_{k}\right)\right]}^{2}=\frac{1}{2}\underset{k}{\sum }{\left[d_{k}-f\left(\underset{j}{\sum }w_{jk}y_{j}\right)\right]}^{2}, \end{array}$$

where *f* is the activation function.

If the function extended to input neurons, where *x*_*n*_ represents the output of the *n*^th^ input neuron and *v*_*nj*_ represents the weight of the connections between the *n*^th^ input neuron and the *j*^th^ hidden layer neuron, then

(4) $$\begin{array}{c} E=\frac{1}{2}\underset{k}{\sum }{\left\{d_{k}-f\left[\underset{j}{\sum }w_{jk}f\left({\text{net}}_{j}\right)\right]\right\}}^{2}=\frac{1}{2}\underset{k}{\sum }{\left\{d_{k}-f\left[\underset{j}{\sum }w_{jk}f\left(\underset{n}{\sum }v_{nj}x_{n}\right)\right]\right\}}^{2}. \end{array}$$

According to the above formula, the total error *E* of the network is the function of every connection weight value *ω*_*jk*_, *v*_*nj*_, so the error *E* can be reduced by adjusting the weight value of connections.

Based on the total error, the optimal weight could be solved by calculating partial derivatives.

(5) $$\begin{array}{c} ∆\omega_{jk}=-\eta \frac{\partial E}{{\partial w}_{jk}},\\ ∆v_{nj}=-\eta \frac{\partial E}{{\partial v}_{nj}}. \end{array}$$

If we do

(6) $$\begin{array}{c} \beta_{k}=\sum \omega_{jk}y_{j},\\ \alpha_{n}=\sum v_{nj}x_{n}, \end{array}$$

then, equation (5) could be written as follows:

(7) $$\begin{array}{c} ∆\omega_{jk}=-\eta \frac{\partial E}{{\partial w}_{jk}}=-\eta \frac{\partial E}{{\partial \beta }_{k}}\frac{{\partial \beta }_{k}}{{\partial w}_{jk}}=-\eta \frac{\partial E}{{\partial \beta }_{k}}y_{j},\\ ∆v_{nj}=-\eta \frac{\partial E}{{\partial v}_{nj}}=-\eta \frac{\partial E}{\partial \alpha_{n}}\frac{\partial \alpha_{n}}{{\partial v}_{nj}}=-\eta \frac{\partial E}{\partial \alpha_{n}}x_{n}. \end{array}$$

After each iteration, the weights were adjusted by adding the change ∆*ω*_*jk*_ or ∆*v*_*nj*_ to the original weights to minimize the total error. A parameter “*η*”, the learning rate, was used to define the weight change along with the gradient descent algorithm. Based on the above formula, the weight change is negative when the gradient is positive and vice versa, which would maintain the solutions towards the least error [39, 48–51].

### 2.3. Search Strategy for Related Studies

In our study, we searched related articles from the following databases: MEDLINE, Embase, Cochrane Library, Chinese Biomedical Literature Database, Wanfang, and CNKI, covering the publish period between January 1, 1966 and May 1, 2019. The search strategy was as follows: “(digestive disease OR digestive system) AND (linear regression OR logistic regression OR logit model) AND (ANN OR back propagation ANN OR BP-ANN) AND (prediction OR diagnostic OR diagnosis).” The titles and abstracts of relevant studies were screened based on eligibility criteria and classified to different groups: (1) duplicated, (2) not relevant, and (3) relevant. Full texts of enrolled studies were assessed by Wei and Yang. Our study was carried out and reported following the recommendations of the Preferred Reporting Items for Systematic Reviews and Meta-Analyses (PRISMA statement) [52].

### 2.4. Selection Criteria for Enrolled Studies

Studies were enrolled if (1) patients were aged from 18 to 65 years and diagnosed with digestive diseases for more than 6 months. Hospital-based or community-based participants were all enrolled; (2) diagnostic or predictive trials were performed compared with linear regression (multiple linear regression, logistic regression, and Poisson regression) and the BP-ANN model simultaneously. The input variables were consistent in linear regression and the BP-ANN model; and (3) outcomes of model accuracy were assessed with following indicators: the area under the receiver operating characteristic curve (AUROC), sensitivity (SEN), specificity (SPE), false-positive rate (FPR), false-negative rate (FNR), and prediction accuracy = (no.of true classified patients/no.of all the patients)∗100% = (SEN + SPE)/(SEN + SPE + FPR + FNR)∗100% [53].

The exclusion criteria were (1) patients who complicated with severe cardiovascular and cerebrovascular disease, (2) patients who have psychological disorder, and (3) patients who suffered malignant digestive tumor and with an expected survival time of less than one year.

The methodological quality of enrolled cohort studies was assessed with the Newcastle-Ottawa quality assessment scale, an established composite score from 3 items: (1) representativeness of exposed and nonexposed patients and the ascertainment of exposure, (2) comparability of cohorts on the basis of the study, and (3) assessment of the outcome and the follow-up was long enough for the outcome to occur.

## 3. Results and Discussion

### 3.1. Characteristics of Included Studies

A total of 319 articles were retrieved from the search strategy, and 43 of them were removed based on screening of titles and abstracts. Two hundred and seventy-six articles were assessed for eligibility and 267 articles were excluded. Nine articles met all the criteria and were enrolled in our review. The flowchart of literature search and the selection process was shown in Figure 3. Of those enrolled articles, the publish year ranged from 1991 to 2017. Seven articles were from China (containing Taiwan Province), one article from Austria, and 1 from Korea. The sample size ranged from 42 to 3222 digestive disease patients, and all of the patients showed comparable biomarkers between the BP-ANN algorithm and linear regression (Table 1).

### 3.2. Diagnosis Accuracy Comparison between the BP-ANN Algorithm and Linear Regression for Digestive Diseases

According to our systematic review, 8 literature demonstrated that the BP-ANN model is superior to linear regression in predicting the disease outcome based on AUROC results (Table 1). Other researchers [63–66] identically demonstrated that the BP-ANN model had great abilities in information processing, high parallelism related to nonlinearity input variables, generalization, and the fault-tolerant capabilities as the nonparametric algorithm, which is widely used for classification, clustering, regression, and dimensionality reduction in several disease fields. The BP-ANN model was superior to linear regression because of its extraordinary processing ability for dealing with the hidden nonlinear relationship between input markers and the clinical outcome, which might be ignored by linear regression and statisticians [67–70].

The self-learning and adaptive capacity of BP-ANN is one of the advantages compared with linear regression [71]. In the two-phase process of training neural networks, the reasonable rules between input and output variables could be automatically extracted through backpropagation self-learning, which would be remembered and then translated to the neuron weights in networks based on adaptive capacity [72–76]. The self-learning phases were commonly repeated for more than 10000 times; the weighted values and error threshold tended to be optimized until the model converges [77]. For most clinicians, a well estimated noninvasive diagnostic model or disease outcome classifier would help to make a correct decision instead of invasive detection. Based on these clinical demands, the BP-ANN training process had the ability to deal with unrecognized confounders for constructing the more accurate classifier, which could transfer training achievements to the unknown information between input variables and clinical outcomes [78–80].

Meanwhile, due to the current availability of big data in multicenter clinical research, enhanced computing power with graphics processing units, and new algorithms to fit neural networks, a computer-aided system could handle thousands of input variables as well as recognize hidden information and made more accurate decisions than fitting in linear regression [81].

The extrapolation performance of the BP-ANN model was a noteworthy development; from the mathematical perspective, BP-ANN could achieve an optimal method that locally searches the global solutions [82–84]. In this process, the weights between neurons were adjusted gradually according to the direction of local improvement, which may enable the algorithm and the weights into local extremum convergence [85]. In addition, BP-ANN was sensitive to initial weights in the network and different initialized networks tend to converge to the related local minimum and many researchers constructed different models after training [79, 86–89].

One literature reported linear regression to be superior to BP-ANN for the early diagnosis of colorectal cancer, in which the input variables were only serum tumor markers, including CEA, CA199, CA242, et al. [46]. Compared with the BP-ANN diagnosis model, logistic regression analysis showed better results, which was related to a multiparameter used within a certain range [90]. The success of the linear regression method in the development of the interpretative and diagnosis model algorithm required the representative and homogeneous of the data structure, elimination of redundancy input variables, appropriate ratio between the number of input variables and the output variables, and accomplishment of strict validation procedures [91–93].

## 4. Conclusions

The noninvasive diagnostic model is one of the vital issues for digestive clinicians and statisticians. Based on our systematic review, the BP-ANN algorithm and linear regression had high capacity in fitting the diagnostic model and BP-ANN displayed more prediction accuracy in most of enrolled studies. To elaborate the situations, we compared the activation functions and data structure between BP-ANN and linear regression for fitting the diagnosis model and the data suggested that BP-ANN was a comprehensive recommendation algorithm.

Based on the traditional three-layer neural networks, statisticians have developed a set of deep learning algorithms with different approaches [94]. Deep learning neural networks (DNN) have extended the depth of layers to four or more layers and performed better than traditional neural networks in diagnosis and prediction when the neural network construction become complex [95–97]. Hinton et al. used an unsupervised restricted Boltzmann machine with deep layers in neural architecture to overcome the limitations of local minimum and overfitting [98]. Also, the convolutional neural network (CNN) encompasses a multilayer of computational connections with minimized processing which performed well in recent research [99–102]. Therefore, further research may focus on the correlations between the traditional neural network and other machine learning algorithms, including deep learning neural networks, convolutional neural networks, and support vector machine method, to select the appropriate algorithm for digestive diseases.

## Figures and Tables

**Figure 1:** The gradient descent of error *E*_*k*_ was calculated for the updated parameters in the BP-ANN algorithm process.

**Figure 2:** The linear regression algorithm process, which was interpreted as the one-layer perceptron neural structure model *Y* = *a* + *b*_1_*x*_1_ + *b*_2_*x*_2_.

**Figure 3:** Flow chart of literature search and the extraction process.

**Table 1:** Characteristics of enrolled studies.

First author	Country	Patient no.	Output marker	Input markers	Algorithm	Results or conclusions
Reibnegger, 1991 [54]	Austria	42	Different liver disease (FL = 1, CPH = 2, and CAH = 3)	Neopterin, AST, ALT, and AST/ALT ratio	Comparison with linear discriminant analysis and with CART and BP-ANN	Compared with the other two techniques, BP-ANN showed a unique ability to detect features hidden in the input data.
Gao, 2004 [55]	China	3222	DM (DM = 1, healthy = 0)	Pulse, family history, nephropathy, waist-to-hip ratio, hypertension, exercise, and age	BP-ANN vs. logistic regression	BP-ANN could assimilate more complicated relationships and is better than logistic regression.
Kim, 2005 [56]	Korea	94	US images of donor liver with respect to macrosteatosis (moderate or severe steatosis = 1, normal or mild steatosis = 0)	ALP, GPT, GOT, *γ*-GGT, hepatorenal ratio of echogenicity, tail area ratio, and tail length of portal vein wall echogenicity	BP-ANN vs. ordinal logistic regression	The area under ROC curve of ANN was significantly greater than that of radiologists (*P* < 0.05).
Liew, 2007 [57]	China (Taiwan)	117	Gallbladder disease (with gallstone = 1, no gallstone = 0)	Gender, age, BMI, waist circumference, hip circumference, SBP, DBP, sugar, CHO, TG, UA, AST, ALT, Alb, WBC, haemoglobin, MCV, insulin, hsCRP, total protein, HDL-C, HbA1C, HOMA, acute inflammation, chronic inflammation, eosinophil, cholesterolosis, cholesterol polyp, and gastric metaplasia	BP-ANN vs. logistic regression	The average correct classification rate of ANNs was higher than that of logistic regression (97.14% vs. 88.2%)
Chuang, 2011 [58]	China (Taiwan)	166	Liver disease (diseased = 1, healthy = 0)	HBsAg, HBeAg, anti-HBs, anti-HBe, anti-HBc, anti-HCV, AST, ALT, TBil, ALB, ALP, r-GT, AFP, gender, marriage, blood type, age, education, occupation, tattoo, smoking, chewing betel nut, alcohol, fatigue, sleep, nap, exercise, breakfast, vegetables, fruits, food date mark, food composition, low salt, healthy status, weight, physical discomfort, healthy examination, acupuncture, and blood donation	A comparison of BP-ANN, CART, logistic regression, and DA	BP-ANN was the best model for liver disease with the accuracy of 95%. The accuracy rates of CART, logistic regression, and DA were 91%, 86%, and 84%, respectively.
Zhang, 2016 [59]	China	120	Pathology diagnosis results of colorectal disease (colorectal patients = 1, benign = 0)	CEA, CA50, HSP60, CYFRA21-1, TPA, AFP, CA199, CA242, CA724, CA125, CA153, and UGT1A8	BP-ANN vs. forward logistic stepwise regression vs. SVM	The AUROC of combined detection was 0.988, in logistic regression. The detection rate was 75% in the BP-ANN model.
Fei, 2017 [60]	China	79	PSMVT (positive or negative)	Age, sex, Hct, PT, FBG, D-dimer, Ca, TG, AMY, APACHEII score, and Ranson score	One-layer BP-ANN vs. logistic regression	The ANN model was more accurate than logistic regression in predicting the occurrence of PSMVT.
Ma, 2017 [61]	China	575	BMI (overweight = 1, healthy = 0)	Weight, height, age, fs-TG, fs-TC, and fs-GLU	BP-ANN vs. multiple linear regression	The BP-ANN models achieved higher prediction accuracy than linear regression.
Shao, 2017 [62]	China	288	Inoperable HCA	Sex, age, stage, diameter, liver metastasis, ascites, prior abdominal surgery, comorbidity, and bismuth stage	BP-ANN vs. logistic regression model	The AUC of the BP-ANN had larger AUC than the multivariate logistic regression model (*P* = 0.02142).

## Data Availability

The data used to support this study could be found in listed references.

## Abbreviations

ANN: Artificial neural network
AUROC: Area under the receiver operating characteristic curve
BP: Backpropagation
CAH: Chronic aggressive non-A, non-B hepatitis
CART: Classification and regression tree
CDC: American Centers for Disease Control and Prevention
CPH: Chronic persistent non-A, non-B hepatitis
DA: Discriminatory analysis
DM: Diabetes mellitus
FL: Fatty liver
FNR: False-negative rate
FPR: False-positive rate
HCA: Hilar cholangiocarcinoma
MSE: Mean square error
PSMVT: Portosplenomesenteric venous thrombosis
PPU: Perforated peptic ulcer
SEN: Sensitivity
SPE: Specificity
TE: Transient elastography
WHO: World Health Organization.
